# Classification of EEG Signal-Based Encephalon Magnetic Signs for Identification of Epilepsy-Based Neurological Disorder

**DOI:** 10.1155/2022/7793946

**Published:** 2022-04-28

**Authors:** Arshpreet Kaur, Suneet Gupta, M. Kathiravan, Syed Nasrullah, Chayan Paul, Saima Ahmed Rahin

**Affiliations:** ^1^GNA University, Village Hargobindgarh, Phagwara, Punjab, India; ^2^Department of CSE, School of Engineering and Technology, Mody University, Lakshmangarh, Rajasthan, 332311, India; ^3^Department of Computer Science and Engineering, Hindustan Institute of Technology and Science, Padur, Kelambaakkam, Chengalpattu 603103, India; ^4^Department of Information Systems, College of Computer Engineering & Sciences, Prince Sattam Bin Abdulaziz University, Al-Kharj, 11942, Saudi Arabia; ^5^Department of Artificial Intelligence and Data Science, Koneru Lakshmaiah Education Foundation, Vaddeswaram, A.P., India; ^6^United International University, Dhaka, Bangladesh

## Abstract

Magnetoencephalography (MEG) is now widely used in clinical examinations and medical research in many fields. Resting-state magnetoencephalography-based brain network analysis can be used to study the physiological or pathological mechanisms of the brain. Furthermore, magnetoencephalography analysis has a significant reference value for the diagnosis of epilepsy. The scope of the proposed research is that this research demonstrates how to locate spikes in the phase locking functional brain connectivity network of the Desikan-Killiany brain region division using a neural network approach. It also improves detection accuracy and reduces missed and false detection rates. The automatic classification of epilepsy encephalomagnetic signals can make timely judgments on the patient's condition, which is of tremendous clinical significance. The existing literature's research on the automatic type of epilepsy EEG signals is relatively sufficient, but the research on epilepsy EEG signals is relatively weak. A full-band machine learning automatic discrimination method of epilepsy brain magnetic spikes based on the brain functional connection network is proposed. The four classifiers are comprehensively compared. The classifier with the best effect is selected, and the discrimination accuracy can reach 93.8%. Therefore, this method has a good application prospect in automatically identifying and labeling epileptic spikes in magnetoencephalography.

## 1. Introduction

Epilepsy is a long-term brain disorder that is caused by brain neurons firing in an unusual way, which causes brain malfunction. In my country, about 3 to 6 percent of people have epilepsy, and intractable epilepsy makes up about 20 percent of that group [1, 2]. There is a 0.02 percent to 0.05 percent growth rate [3].

When it comes to cognitive neuroscience, sFC has become an important tool. A study called “spontaneous functional connectivity” looks at the statistical relationships between spontaneous fluctuation signals in different parts of the brain, and some studies say it can show how the brains of different parts of the brain work together [4]. There are two basic components of the brain, and these brain components are nodes and edges. The nodes and edges play an important role to indicate distinct brain areas, while the boundaries depict the connection between them. The edges are used to determine how functionally connected nodes are. But nodes indicate a predetermined group of the central nervous system. As a tool for neuroscience research, spontaneous functional connectivity can help us learn more about how the brain works outside of a specific task [5, 6]. An important and widely used tool called “spontaneous functional connectivity” can be used to find out how the brain works and how it works normally. It can also be used to show how the brain works in different types of neurological and psychiatric disorders like strokes, Parkinson's, Alzheimer's, epilepsy, and autism.

Using data from magnetic resonance imaging (fMRI), Biswal found that blood oxygenation changes were caused by natural fluctuations in the network. The same network was also found in brain electrophysiological recordings like EEG and magnetoencephalography [5, 7]. Many studies use fMRI because it has a high level of spatial resolution. Another problem with this method is that its low temporal resolution (0.5–2 Hz) and vessel-based contrast make it impossible to directly study high frequencies, which are thought to be the information exchange mechanism between brain regions, called neocortical activity [7]. As a result, the time scale of neural activity is usually much faster than the recording speed of fMRI [8].

A noninvasive method called magnetoencephalography (MEG) is used to measure the magnetic field that is caused by the activity of nerve bundles. Because of its sampling rate, it can look at fast brain activity right away [9]. MEG was used in this study to get a wide range of neurophysiologically relevant frequency bands because it has a very high temporal resolution. In addition, a number of studies have shown that phase relationships between cortical regions can be used to measure functional connectivity. This is especially true of the phase locking value, which measures the phase synchronization between two time series. This was previously used to look at the resting-state connection between the MEG and the brain. The magnetoencephalography (MEG) is already widely used in clinical examinations and medical research. The brain network approach that is based on resting-state magnetoencephalography could be utilized to examine normal or abnormal brain functions. In addition, magnetoencephalography analysis provides a high reference value for epilepsy diagnoses.

Connect with each other to build a brain functional network. So, magnetoencephalography is an important way to help with the diagnosis of epilepsy. Epilepsy is a progressive neurodegenerative illness wherein brain function gets unbalanced, resulting in convulsions or episodes of strange behavior, feelings, and even absence of consciousness. We can learn more about how the brain operates outside of a given activity by studying spontaneous functional connectivity. In magnetoencephalography, the main signs of epilepsy are spikes and sharp waves, but sometimes, they are not separate and are called epilepsy transients [10] or spikes. They stand out from the rest of the activity because they have higher amplitudes and last for 20 to 200 ms.

Doctors look at patients' magnetoencephalograms and look for signs of abnormal brain activity, which they do by looking at them and analyzing them based on their own experience. There are a lot of things that do not go well with visual inspection. Most of the time, it takes 60 minutes to record the data for a single review. It takes a lot of work to find spikes in very long data, and the analyst has to be very careful. Many people who have epilepsy cannot be sure that classification results will be accurate when they have a lot of work to do. Furthermore, different experts look at the same record in a different way. So, the automatic detection of abnormal brain electrophysiological signals is very important [11]. Spontaneous functional connectivity is a technique for neuroscience study; spontaneous functional connectivity can teach us all about how the brain functions when it is not doing a specific activity. It may also be used to demonstrate how the brain functions in various neurological and mental illnesses such as injuries, Parkinson's, Alzheimer's, epilepsy, and autism. All the time, it is important that the spike wave detection results have a higher correct rate and less missed detection and false detection. This paper shows how to use a machine learning method to look for spikes in the Desikan-Killiany brain area division's phase-locked brain functional connectivity network to find them. Automatically identifying and marking epilepsy spikes help doctors do less work, improve detection accuracy, and reduce missed and false detection rates. An auxiliary tool for this helps doctors do less work and improve detection accuracy.

The present article has been planned into five sections.  Section 1 describes the introduction of the proposed research, the data and methods are described in Section 2, Section 3 puts light on model design, the experimental results and analysis of the proposed research are described in Section 4, and finally, Section 5 portrays the conclusion and possible future-based work on the proposed framework.

## 2. Data and Methods

### 2.1. Data Collection

The MEG data used in this article were obtained from 20 patients diagnosed with epilepsy in the insular lobe and insular cap, examined by the Magnetoencephalography Center of Xuanwu Hospital of Capital Medical University, 15 to 52 years old, with an average of 28.7 years old.

For MRI, 1.5 T or 3.0 T was used for standard MRI scans, including transverse SE sequence T1W1 and TSE sequence T2W1 (slice thickness 5 mm), with oblique coronal view perpendicular to the long axis of the right hippocampus and transverse view parallel to the long axis of the hippocampus, using fluid-attenuated inversion recovery (FLAIR) sequence (slice thickness 5 mm).

MEG uses the NM20215A-G 306-channel full-head biomagnetism instrument produced by Elekta Neuromag Oy in Finland to detect patients. The patients recorded spontaneous magnetoencephalography data for 60 min in a magnetically shielded room in a calm state. The band-pass filtering is 0.10~330 Hz, and the sampling rate is 1000 Hz. Magnetic brain imaging (MSI) was acquired by a standard procedure 306-lead whole-head magnetoencephalography system, and the interracial epileptiform waves were labeled and analyzed offline. Magnetic brain waves are fused with patient MRI images to generate MSI images on the MRI automatically.

The doctor of the magnetoencephalography center selects three data segments containing spike waves for each case based on experience; each piece is 10 s each and marks the time point of the spike wave peak value; as a comparison, three regular components are provided for each case. First is the resting-state data segment; each piece is 10 s; to ensure the correctness and typicality of the spike wave data selected this time and the average resting-state data, different doctors were specially invited to conduct cross-check confirmation to ensure that the two kinds of data used in this study are typical spike wave state and typical average resting-state magnetoencephalography data.

### 2.2. Data Preprocessing

After obtaining the MEG data of all 20 cases selected by doctors using traditional methods, the MEG analysis software Brainstorm (brain recordings analysis tool) based on the mathematical software Matrix Laboratory (MATLAB) platform was used for data preprocessing. First, the MEG is filtered to obtain the data in the 0.1-500 Hz frequency band; then, the artifacts in the data are removed, including the interference of electrooculography and eye movement, for MEG.

After all the data were processed in strict accordance with the above method, the data segment with a spike wave peak value of 2000 ms was intercepted from the 10 s data segment with spike waves provided by the doctor, and the data of the same length was blocked from the middle of the 10 s spike-free data segment. Finally, a total of 2000 ms long data segments with spikes and 60 data segments without points were obtained, and these data are the bases for further analysis.

### 2.3. Establishment of Brain Functional Network

All data were automatically analyzed and processed through the Ubuntu platform-based workstation, called the Free Surfer software package. The analysis and processing process is divided into two parts: volume processing process and surface processing process. The volume processing pipeline includes image greyscale normalization, correction of nonuniform magnetic fields, registration to Talairach space, removal of nonbrain tissue, and segmentation of white matter (WM) and grey matter (GM). The distance between the grey matter surface and the white matter surface was defined as the thickness of the cerebral cortex, and the *T*-average method is used to determine the thickness of the cortex. The grey matter's outermost layers grow outward, creating an elevated surface. The inflating surface is recorded with the templates in a high dimension after spherical distortion, and the cortex is autonomously divided as per the Desikan-Killiany map. The surface treatment process includes a three-dimensional reconstruction of the white matter surface, starting from the white matter surface and expanding outward along the grey matter gradient to obtain the grey matter outer surface. The distance between the grey matter surface and the white matter surface was defined as the thickness of the cerebral cortex, and the *T*-average algorithm was used to calculate the thickness of the cortex. The outer surface of the grey matter expands outward, resulting in a raised surface. After spherical deformation, the inflation surface is registered with the template in a high dimension, and the cortex is automatically partitioned according to the Desikan-Killiany map. The Desikan-Killiany atlas divides the whole brain into 70 brain regions (35 in each of the left and right hemispheres), in which the corpus callosum has no grey matter thickness, so the cortical thickness of 68 brain regions (34 in each of the left and right hemispheres) is finally obtained. All data were sourced by the Dipole method in Brainstorm software, and then, the sourced data of each case and each band were downsampled according to the Desikan-Killiany map. The volume processes process and surface processing process start with the white matter surface and spread outwards and along the grey matter volume curve to acquire the grey matter outer surface; the surface treatment method comprises a three-dimensional reconstruction of the white matter surface. The width of the cerebral cortex was calculated using the *T*-average technique, and the gap between the grey and white matter surfaces was designated as the width of the cortex.

The two most basic and critical components of a brain network are nodes and edges: nodes represent various brain regions, and borders reflect the connections between different brain regions. For example, the 68 brain regions divided by the Desikan-Killiany template are defined as nodes in the brain network, as shown in Figure 1; each brain region is a node.

Phase locking value (PLV) is used to build brain functional networks [12, 13]. The phase locking value shows how likely it is for two time series signals to stay in the same phase over a period of time. Using electrophysiological recordings, it is possible to figure out how the phase difference between two time series at a given frequency changes over time. This is called “resting-state phase locking.” The formula for figuring out PLV looks like this:

(1) $$\begin{array}{c} \text{PLV}=\frac{1}{N}\left|\overset{N}{\underset{n=1}{\sum }}e^{i\left(\theta_{1}\left(n\right)-\theta_{2}\left(n\right)\right)}\right|. \end{array}$$

Among them, *N* is the number of sampling points, *θ*_1_ and *θ*_2_ are the instantaneous phase values at sampling point *n*, and the phase locking value is a complex number whose modulus ranges from 0 to 1, where 0 represents a random phase relationship, and 1 represents a fixed phase relation. Phase locking is a measure that does not go in any direction, so it is symmetrical. Each time two cortical brain area time-series measurements are made, the whole-brain phase locking network is calculated between each pair of measurements. To figure out phase locking values between time series measurements, you only need to figure out one value for each pair of time-series measurements because phase locking is square.

After downsampling, the data of each source is obtained. The phase locking value plays an important role in the brain functional network. It indicates whether likely two time series signals are to remain in the same aspect throughout a period. It is important to calculate how the phase gap between two sequences at a particular frequency changes with time. Then, the phase locking value (PLV) matrix is obtained for all individual data segments in all two groups of data in the frequency range of 0.1~500 Hz and divided into seven frequency bands. The corresponding frequency ranges of all seven frequency bands from the low frequency of F1 to the high frequency of F7 are shown in Table 1.

The phase locking value matrix in a single frequency band is randomly selected as a typical display for representativeness. Here, the phase locking value matrix of the 2000 ms data segment in the alpha frequency band of Case No. 3 is selected and shown in Figure 2.

## 3. Model Design

This paper uses three traditional classification algorithms: linear logistic regression classification, support vector machine classification based on linear kernel function and radial basis kernel function, and Gaussian Naive Bayes classification algorithm. The above models are implemented using parts under the scikit-learn framework.

### 3.1. Linear Classification

This paper uses the sigmoid function as the linear logistic regression (logistic regression) classifier function. The sigmoid function is the most widely used class of classification functions, which is defined as

(2) $$\begin{array}{c} y=\frac{1}{1+\exp\left(wx+b\right)}. \end{array}$$

Among them, *y* is the probability that the sample is positive and 1 − *y* is the probability that the piece is negative. To ensure the training accuracy of the model, the loss function introduces the L1 regularization term, in which the reciprocal of the regularization coefficient *C* = 1.0 is set, and the model predicted value is the probability value of the binary classification. The loss function is

(3) $$\begin{array}{c} l={\left\|w\right\|}_{1}+C\overset{n}{\underset{i}{\sum }}\ln\left(\exp\left(-y_{i}\left(X_{i}^{T}w+b\right)\right)+1\right). \end{array}$$

Calculate the parameters (*w*, *b*) when the loss function takes the minimum value; that is, you can get the optimal classification model.

### 3.2. Support Vector Machine

Support vector machines construct a hyperplane or a series of hyperplanes in a high-dimensional or infinite-dimensional space and use the hyperplane to achieve segmentation to maximize the gap between positive and negative samples. The model has a good effect on nonlinear relationship classification. The basic principle is as follows.

Given a training vector *x*_*i*_ ∈ *R*^*P*^, *i* = 1, 2, 3, ⋯, *n*, and a label vector *y* ∈ {1,−1}^*n*^. There is a hyperplane *w*^*T*^ *x* + *b* = 0 in the sample space to effectively classify the samples; there are

(4) $$\begin{array}{c} \left\{\begin{array}{c} w^{T}\cdot x+b\geq +1,\;y=+1,\\ w^{T}\cdot x+b\leq -1,\;y=-1. \end{array}\right. \end{array}$$

The points closest to the hyperplane for which equation (4) is established constitute a support vector. The sum of the distance from the support vectors in the forward and reverse directions to the hyperplane is *γ* = 2/‖*w*‖. The parameter that minimizes the space is the optimal parameter. Using $\underset{w,b}{\min}1/2{\left\|w\right\|}^{2}$ as the objective function of the formula, the optimization is carried out according to the Lagrange multiplier method, which is simplified to the dual problem:

(5) $$\begin{array}{c} \underset{a}{\max}\overset{m}{\underset{i=1}{\sum }}\alpha_{i}-\frac{1}{2}\overset{m}{\underset{i=1}{\sum }}\overset{m}{\underset{j=1}{\sum }}\alpha_{i}\alpha_{j}y_{i}y_{j}x_{i}^{T}x_{j}\\ \text{s}.\text{t}.\overset{m}{\underset{i=1}{\sum }}\alpha^{i}y^{i}=0,\;\alpha^{i}\geq 0. \end{array}$$

When the original spatial hyperplane cannot effectively separate the data, it must map it to a high-dimensional space, i.e., *x* ↦ *φ*(*x*). In the dual problem, find the kernel function *κ*(*x*_*i*_, *x*_*j*_) such that *κ*(*x*_*i*_, *x*_*j*_) = {*φ*(*x*_*i*_), *φ*(*x*_*j*_)} = *φ*(*x*_*i*_)^*T*^*φ*(*x*_*j*_), in order to realize *φ*(*x*_*i*_)^*T*^*φ*(*x*_*j*_) inner product calculation. This paper adopts linear kernel function (kernel:linear) and radial basis kernel function (kernel:rbf).

### 3.3. Naive Bayesian Classification

The Naive Bayesian classifier (NBC) has been widely used due to its high computational efficiency, high accuracy, and solid theoretical foundation. The Bayesian classifier uses the Bayesian equations to determine the likelihood of a label based on the likelihood of a brand. The class with the highest conditional distribution is then chosen as the class whereby the item would belong.

In general, all attributes in Bayesian classification play a role directly or indirectly; that is, all details participate in the category, rather than one or several points determining the type [14]. The Bayesian classifier uses the Bayesian formula to figure out the probability of a label through the chance of a brand. Then, it chooses the class with the highest posterior probability as the class to which the object should belong. Any two pairs of features are not connected to each other, and you should think that each sample is unique and distributed the same way across all of them. Then, according to the central limit theorem, the data of each part after normalization satisfies the assumption of Gaussian distribution, that is, *P*(*x*_*i*_ | *y*) ~ Gaussian; according to Bayes' theorem, we have

(6) $$\begin{array}{c} P\left(y\left|x_{1},x_{2},\cdots ,x_{n}\right.\right)=\frac{P\left(y\right)P\left(x_{1},x_{2},\cdots ,x_{n}\left|y\right.\right)}{P\left(x_{1},x_{2},\cdots ,x_{n}\right)}. \end{array}$$

According to the assumption that each pair of features is independent of each other, there are

(7) $$\begin{array}{c} P\left(y\left|x_{1},x_{2},\cdots ,x_{n}\right.\right)\propto P\left(y\right)\overset{n}{\underset{i=1}{\prod }}P\left(x_{i}\left|y\right.\right). \end{array}$$

The posterior distribution of *y* can be calculated according to equation (7).

### 3.4. Original Feature Construction

C2 was selected at each frequency band based on the symmetry of the relationship among the 68 cortical regions. 68 independent sets of data of 7 frequency bands form a 15 946-dimensional vector. According to the corresponding method of each group of features, 120 sample data (including 60 average resting state sample data and 60 spike wave state sample data) are combined to form a 120 × 15 946 dataset. These data constitute the original feature space, and 40% of the randomly selected dataset is divided into the test set, and the remaining 60% is divided into the training set.

In the research, the PLV complex matrix data itself (plv) as the original feature space, the fundamental part (plv_real), the imaginary part (plv_imag), the argument (plv_angle), and the modulus (plv_abs) of the matrix data were tested, respectively. The results show that of all the models used, the modulo data performs the best. Taking the Naive Bayes classifier model as an example, the accuracy of the five-item data classification is shown in Table 2.

After testing, the above five data have similar performance to the other four classifier models used in this paper, so the data mentioned in this paper are the modulo (plv_abs) data of the PLV complex number matrix, and the original feature space complex number matrix is selected. The modulo data is used as the original feature dataset. The above four classifiers are used in the experiment to learn and classify the plv_abs data, respectively. The experimental results are shown in Table 3.

## 4. Experimental Results and Analysis

### 4.1. Experimental Procedure

Firstly, the original feature dataset of 120 × 15 946 was used as input. Then, the input dataset was standardized. Finally, three chi-squared tests, *F* tests, and iterative feature elimination were applied to the standardized dataset for feature extraction; four classifiers were used to classify the above data, and all the experimental results were analyzed and compared. The processing flow after the original feature dataset is constructed is shown in Figure 3.

### 4.2. Experimental Results

To compare the various approaches qualitatively, this paper compares the Receiver Operating Characteristic (ROC) curve plots of the four classifiers. The ROC curve is a comprehensive indicator reflecting true positives and false positives. The predictions of the four classifiers in this paper are all probability values. The spike wave is marked as a positive example, and the intermediate state without a spike wave is unfavorable. Sort the test results according to the probability value of the positive model, and then use different probability values as the threshold for positive and negative examples, and calculate the actual positive rate and false positive rate under the corresponding entry. Then, the ROC curve of the classifier can be drawn. Generally, according to the different requirements of the classification task, there are different standards for evaluating the classifier's performance according to the curve. The ROC curve of the classifier in this paper is crossed. The four classifiers in this paper's projections are all probabilistic values. A good example is the spike wave, while the transitional condition without the need for a spike wave is undesirable. Arrange the test results according to the positive model's significance level. Therefore, this paper uses the general AUC (area under the ROC curve) method to evaluate the classifier's performance. To evaluate, AUC is the part area enclosed by the ROC curve and the axis. The larger the size, the better the classification performance of the classifier.

### 4.3. Experimental Comparison of Original Feature Datasets

Using the plv_abs data as the initial feature dataset input, after training the four classification models, the experimental results are shown in Table 3 and Figure 4.

It can be seen from Table 3 and Figure 4 that the accuracy of the Naive Bayes classifier model is 0.875, which is higher than the other three models, and its AUC value is 0.914, which is also the second-highest among all classifiers. For raw data, the SVM classifier with linear kernel function performed best.

### 4.4. Experimental Comparison of Feature Normalization

The feature vector data of each column of the original feature dataset are standardized according to

(8) $$\begin{array}{c} x_{\text{std}}=\frac{x_{i}-\mu_{i}}{\sigma_{i}}. \end{array}$$

Among them, *x*_*i*_ represents the *i*th feature vector, *σ*_*i*_ represents the standard deviation of the feature in this column, *μ*_*i*_ represents the mean of the *i*th feature, and *x*_std_ represents the normalized feature vector.

Using the normalized data as input, after training the four models, the test results are shown in Table 4 and Figure 5.

After normalizing the data of each column of the original training set, the accuracy of the linear logistic regression classifier improved from 0.771 to 0.917. The major benefits of the support vector machine are that it has a good effect on nonlinear relationship classification. The radial basis kernel function support vector machine classifier that would have been chosen has the maximum benefit on automated spike categorization. The accuracy of the support vector machine classifier using the linear kernel function improved from 0.833 to 0.917 and the radial accuracy rate of the basis kernel function support vector machine classifier.

The improvement from 0.500 to 0.938 indicates that the progress is the highest. The accuracy of the Naive Bayes classifier is also slightly improved from 0.875 to 0.896, meaning that standardizing each column's data of the original training set is conducive to improving the accuracy. For the four classifiers, the performance is not much different in terms of accuracy, and the combination is used as a score.

For the AUC value of the performance evaluation standard of the classifier, the AUC value of the radial basis kernel function support vector machine classifier is 0.951, which is the largest among the four classifiers. Therefore, the standardized feature dataset is used as the input based on the above results. The selected radial basis kernel function support vector machine classifier has the best effect on the automatic classification of spikes, with a success rate of 93.8%.

#### 4.4.1. Feature Extraction

The existence and related effects of spike waves can be easily identified based on empirical knowledge in actual human identification. However, the observation and judgment of 15 946-dimensional data cannot be realized in a short time. The procedure of translating primary converted into static characteristics which can be analyzed while keeping the information from the source dataset is known as feature extraction. Filtering based on multivariate analytical techniques is used to extract the features. Therefore, it is inferred that there must be a large number of redundancy, so feature selection is performed based on appropriate tolerance of model performance degradation to reduce the complexity of the model.

*(1) Feature Selection Based on Univariate*. Features are selected by filtering based on univariate statistical tests. In this paper, the chi-squared test and *F* test method are used to test the correlation between individual characteristics and experimental labels one by one and select some features according to the correlation ranking. Based on multiple tests of the extracted features, it is determined that 32 components are chosen; that is, 0.2% of the total number of elements can achieve high classification accuracy and significantly reduce the number of features. The 32 components extracted by the *F* test and the chi-squared test are inconsistent.

*(2) Model-Based Recurrent Feature Elimination (RFE)*. In this paper, a logistic regression classification model is adopted, L1 is used for regularization, and 32 features are selected.

#### 4.4.2. Experimental Comparison of Data after Feature Selection

The 32 feature vectors screened by the three feature selection methods were used as input, and after training the four classification models, the experimental results are shown in Table 5 and Figures 6–8.

It can be seen from Tables 5 and 6 that after the feature selection by the iterative feature elimination method, the classification accuracy and AUC value of the classifiers under the four classifiers are lower than those of the other two selection methods, indicating that in this kind of feature, the effect of the selection method is not good, so focus on the chi-squared test and the *F* test feature extraction selection method.

Compared with the experimental results after feature standardization, the accuracy of the linear logistic regression classifier was reduced from 0.917 to 0.833 and 0.833; the accuracy of the linear kernel function support vector machine classifier was decreased from 0.917 to 0.896 and 0.792, while in the radial basis kernel function, the accuracy rate of the support vector machine classifier is reduced from 0.938 to 0.833 and 0.854, indicating that after feature selection, using the above three classifiers for classification, the accuracy rate will be diminished, and for the Naive Bayes classifier, using the chi-squared test and *F* test feature extraction data as input, the accuracy rate increased from 0.896 to 0.917, which is the classifier.

The AUC value has increased from 0.912 to 0.951, which is higher than that of the other three classifiers, indicating that the Naive Bayes classifier has the best performance and the best classification for the chi-squared test and *F* test feature extraction effect.

## 5. Conclusions

The 18 key feature positions listed in this paper are restored and calculated, and the positions obtained are (1, 20) (1, 22) (1, 60) (9, 13) (12, 20) (15, 31) (15, 65) (18, 33) (18, 48) (18, 52) (25, 42) (28, 38) (30, 61) (30, 62) (31, 38) (32, 54) (55, 66) (59, 65); 18 features are all in the delta band. If we compare the proposed method with existing methods, the proposed method is more capable because it automatically identifies and classifies epileptic spikes in magnetoencephalography; it might be a potential approach for this technology. Therefore, it can be concluded that the EEG signal that determines epilepsy can be completely discriminated by the signal in the delta frequency band. The future scope of this research is that it will play a crucial role in future studies. The proposed approach has a good application prospect in automatically identifying and labeling epileptic spikes in magnetoencephalography. One of the major drawbacks of EEG is that it is difficult to determine where in the brain the neural impulse is originating from. It is suggested that in the follow-up medical practice, the signal transmission between the 18 pairs of cerebral cortical regions corresponding to the above 18 characteristics should be focused on, and the next step would be to carry out research on the above brain regions in clinical practice.

## Figures and Tables

**Figure 1:** Partition map of 68 brain regions in the whole brain.

**Figure 2:** Phase locking value matrix.

**Figure 3:** Experimental flow chart.

**Figure 4:** ROC plots of raw data.

**Figure 5:** ROC plots of normalized raw data.

**Figure 6:** Comparison of learning classification ROC based on chi-squared test to extract features.

**Figure 7:** Comparison of learning classification ROC based on *F* test feature extraction.

**Figure 8:** Comparison of learning classification ROC based on features after iterative feature elimination.

**Table 1:** Band correspondence table.

Band number	Band name	Frequency range (Hz)
F1	Delta	0.1~3
F2	Theta	4~7
F3	Alpha	8~12
F4	Beta	15~29
F5	Gamma1	30~59
F6	Gamma2	60~80
F7	Ripple	81~250

**Table 2:** Accuracy distribution table based on Naive Bayes classifier model.

Data	Classification accuracy
plv	0.444
plv_real	0.444
plv_imag	0.472
plv_angle	0.417
plv_abs	0.917

**Table 3:** Comparison of classification accuracy and AUC results of different models based on original data.

Model	Raw feature data accuracy	AUC
Logistic regression	0.771	0.716
SVC_linear	0.833	0.985
SVC_RBF	0.500	0.854
Gaussian NB	0.875	0.914

**Table 4:** Comparison of classification accuracy and AUC results of different models based on standardized data.

Model	Standardized feature data accuracy	AUC
Logistic regression	0.917	0.914
SVC_linear	0.917	0.903
SVC_rbf	0.938	0.951
GaussianNB	0.896	0.912

**Table 5:** Comparison of classifier accuracy under different feature selection methods.

Model	Chi-squared test to extract features	*F* score to extract features	Data after iterative feature removal
Logistic regression	0.833	0.833	0.750
SVM (kernel:linear)	0.896	0.792	0.750
SVM (kernel:rbf)	0.833	0.854	0.833
GaussianNB	0.917	0.917	0.875

**Table 6:** AUC comparison of each model under different feature selection methods.

Model	Chi-squared test to extract features	*F* test to extract features	Data after iterative feature removal
Logistic regression	0.905	0.914	0.845
SVM (kernel:linear)	0.965	0.878	0.854
SVM (kernel:rbf)	0.951	0.938	0.907
GaussianNB	0.951	0.951	0.919

## Data Availability

The data shall be made available on request.

## References

[1] Frolov N. S., Hramov A. E. Multilayer perceptron reveals functional connectivity structrure in thalamo-cortical brain network.

[2] Neşe H., Bayram A., Harı E., Kurt E., Ademoğlu A., Demiralp T. Phase consistency analysis of the brain functional connectivity networks.

[3] Yuan Y., Wang Y., Chen X., Wei F. Inferring human brain structural connectivity based on neural networks.

[4] Li H., Satterthwaite T. D., Fan Y. Brain age prediction based on resting-state functional connectivity patterns using convolutional neural networks.

[5] Ratta P., Kaur A., Sharma S., Shabaz M., Dhiman G. (2021). Application of blockchain and Internet of things in healthcare and medical sector: applications, challenges, and future perspectives. *Journal of Food Quality*.

[6] Marui W., Kan S., Nii M., Shibata M., Kobashi S. MD-LMS algorithm based brain functional connectivity analysis in resting state fMRI.

[7] Shiba K., Kaburagi T., Kurihara Y. A dynamic Bayesian network analysis of functional connectivity during a language listening comprehension task.

[8] Chopra S., Dhiman G., Sharma A., Shabaz M., Shukla P., Arora M. (2021). Taxonomy of adaptive neuro-fuzzy inference system in modern engineering sciences. *Computational Intelligence and Neuroscience*.

[9] Baselli G., Bergsland N., Costantini I. Integrating structural and functional brain connectivity image, signal, and data processing problems.

[10] Tiwari A., Dhiman V., Iesa M. A. M., Alsarhan H., Mehbodniya A., Shabaz M. (2021). Patient behavioral analysis with smart healthcare and IoT. *Behavioural Neurology*.

[11] Huang J., Zhou L., Wang L., Zhang D. (2020). Attention-diffusion-bilinear neural network for brain network analysis. *IEEE Transactions on Medical Imaging*.

[12] Rangaprakash D. (2017). Binarized brain connectivity: a novel autocorrelation-based iterative synchronization technique. *IEEE Transactions on Signal and Information Processing over Networks*.

[13] Roland G., Kumaraperumal S., Kumar S., Gupta A. (2021). PCA (principal component analysis) approach towards identifying the factors determining the medication behavior of Indian patients: an empirical study. *Tobacco Regulatory Science*.

[14] Miller R. L., Calhoun V. D. Transient spectral peak analysis reveals distinct temporal activation profiles for different functional brain networks.

